# Effects of Stress on Osteoblast Proliferation and Differentiation Based on Endoplasmic Reticulum Stress and Wnt*β*-Catenin Signaling Pathway

This article has been retracted.

**DOI:** 10.1155/2022/8521051

**Published:** 2022-09-19

**Authors:** Hanming Zhong, Xiaoyu Yang, Shitie Li, Xin Lei

**Affiliations:** ^1^Stomatology Department, Affiliated Dongguan Hospital, Southern Medical University (Dongguan People's Hospital), Dongguan, Guangdong 523000, China; ^2^Center of Oral Implantology, Stomatological Hospital,Southern Medical University, Guangzhou, Guangdong 510280, China; ^3^Department of Stomatology, Shenzhen Longhua District Central Hospital, Shenzhen, Guangdong 518110, China

## Abstract

In order to investigate the effect of fluid shear stress on the proliferation of osteoblasts and the regulatory role of the Wnt/*β*-catenin signaling pathway in cell proliferation, a new method based on endoplasmic reticulum stress and Wnt/*β*-catenin signaling pathway stress-mediated was proposed. Taking MG63 osteoblasts as the research object, they were inoculated on glass slides (G group), polished titanium sheets (P group), and sandblasted acid-base treated pure titanium sheets (S group). In addition, FSS of 0 dunes/cm^2^ (static group) and 12 dunes/cm^2^ (stress group) were given, respectively. Then, quantitative reverse transcription-PCR (RT-qPCR) and western blot were used to detect the mRNA and protein expressions of low-density lipoprotein receptor-related protein 5 (LRP5) and *β*-catenin in MG63 cells. The results showed that the expression levels of *β*-catenin mRNA and protein in cells in the stress group were significantly increased (*P* < 0.05), and the protein expression level of LRP5 was significantly decreased (*P* < 0.05). The expression level of LRP5 in group *S* was greatly inhibited, while the expression level of *β*-catenin was significantly upregulated. Therefore, FSS can stimulate the expression of LRP5 and *β*-catenin in osteoblasts. Fluid shear stress can promote osteoblast proliferation in vitro; the Wnt/*β*-catenin signaling pathway is involved in regulating fluid shear stress to promote osteoblast proliferation.

## 1. Introduction

Implant denture has gradually become an important trend in the repair of dentition defects and loss, and the success rate of clinical application is high, but there were some individual failure cases [1]. The success of implant dentures depends on whether good osteosynthesis can be achieved. The dynamic balance between the osteogenic effect of osteoblasts and the bone resorption of osteoclasts plays a decisive role in the process of bone healing, and it is also closely related to biomechanics and other factors [2, 3]. At present, most studies mainly use two-dimensional or three-dimensional finite element analysis to explore the influence of dental force transmissions, such as jaw bone quality, implant morphology, and dental force [4, 5]. However, there are relatively few studies on biomechanical transduction and biological effects of implant interface.

Among all the stresses, mechanical tension and flow shear stress (FSS) are the most important forces on the implant-bone interface [6]. There is a large amount of reticulated bone cancellous in bone tissue, and the pressure of tissue or the pulse of blood vessels can cause the flow of interstitial fluid in bone trabeculae and then produce FSS on bone tissue cells [7]. Under the action of mechanics, the effect of cellular resistance will undergo corresponding morphological changes, accompanied by a series of signal pathway activation or inhibition [8]. Present studies showed that the low-density lipoprotein receptor-associated protein 5 (LRP5) in the Wnt signaling pathway is closely related to the progression of osteoporosis [9]. Moreover, many studies suggested that LRP5 is closely related to bone metabolism [10–12]. However, it is still unclear whether the Wnt signaling pathway can participate in the biomechanical signaling process.

Therefore, the expression changes of Wnt/beta-catenin scanning signaling pathway-related mRNA and protein in MG63 cells after FSS treatment were analyzed. The purpose of this study was to investigate the effects of the Wnt signaling pathway and biomechanics on osteoblast activation and to provide more evidence for biomechanical studies of implant-bone interface cells.

## 2. Materials and Methods

### 2.1. Test Materials

MG63 cells were purchased from ATCC, USA. TA0 grade Shengye pure titanium plate was purchased from Shaanxi Baoji three-line Nonferrous Metal material factory. BCIP/NBT alkaline phosphatase color reagent kit was purchased from Shanghai Beyotime Biotechnology Co., Ltd. Alizarin Red was purchased from Shanghai Beyotime Biotechnology Co., Ltd. Trizol reagent total RNA extraction kit was purchased from Invitrogen, USA. The RNA reverse transcription kit was purchased from Invitrogen, USA. SYBR Green I detection kit was purchased from Invitrogen, USA. Dulbecco's modified Eagle's medium (DMEM) low-sugar medium was purchased from Hangzhou Genom Company. Fetal bovine serum was purchased from Gibco, USA. Penicillin and streptomycin were purchased from Hyclone, USA. The nuclear protein extraction kit was purchased from Merck, Germany. Rabbit antihuman LRP5 antibody was purchased from a cell signaling technology company, USA. Rabbit antihuman *β*-catenin antibody was purchased from a cell signaling technology company, USA. Rabbit antihuman *β*-actin antibody and rabbit antihuman *α*-tubulin antibody were purchased from Shanghai Beyotime Biotechnology Co., Ltd.

### 2.2. Culture of Osteoblasts

MG63 osteoblasts were cultured in a DMEM medium containing 10% fetal bovine serum and 1% penicillin-streptomycin, respectively and placed in a 37°C incubator containing 5% CO_2_ and 100% humidity. The cell culture medium was replaced every 48 h. When the confluence of cells reached about 80%, the cells were digested with 0.25% trypsin, and the cells were subcultured. After a 3–4 d culture, FSS treatment was performed.

### 2.3. Preparation of Titanium Surface and Self-Made Steady Flow Loading System

The rectangular specimen with a length of 75 mm, a width of 25 mm, and a thickness of 1 mm was processed by pure titanium plate wire cutting. Smooth slides of the same size were used as the control group, which were rolled into polishing treatment and sandblasting-acid and alkali treatment according to the processing methods. They were named group G, group P, and group S, respectively, and their surface morphology was observed by scanning electron microscopy.

The flow chamber system designed by Hochmuch et al. [13] was referred to as a blueprint for manufacturing. The entire fluid loading system is mainly composed of a peristaltic pump, a silicone tube, a liquid storage bottle, a buffer bottle, and a flat flow chamber. A precision peristaltic pump provides an FSS of 12 dunes/cm^2^. After being pumped from the peristaltic pump, the perfusion fluid enters the flow cavity through the pipeline, applies corresponding shear stress to the cells, and then enters the liquid storage bottle through the pipeline, thereby forming a closed circulation system.

### 2.4. Real-Time Fluorescence Quantitative PCR Detection

Cells after stress were rolled into 0 dynes/cm^2^ (stationary group) and 12 dynes/cm^2^ (stressed group). Primary osteoblasts and MG63 osteoblasts were collected at 0 h, 0.25 h, 0.5 h, 1 h, 2 h, and 4 h after stress. Trizol reagent was used to extract total RNA from cells, and the purity and concentration were detected. cDNA reverse transcription was carried out according to the cDNA reverse transcription kit, and the products were stored at −20°C for later use. Primers for quantitative detection of LRP5 and *β*-catenin mRNA sequences were designed and synthesized, and the specific information is shown in Table 1. RT-qPCR kit was used for quantitative detection of target gene mRNA levels in cells.

### 2.5. Western Blot

MG63 osteoblasts were collected and lysed at 0 h, 0.25 h, 0.5 h, 1 h, 2 h, and 4 h after stress and total protein was extracted. The standard curve of the extracted protein concentration was drawn using the BCA protein concentration detection kit, so as to carry out the quantitative detection of the sample protein. 10% sodium dodecyl sulfate-polyacrylamide gel electrophoresis (SDS-PAGE) adhesive was configured, and electrophoretic separation of proteins was performed after sample loading. At the end of electrophoresis, the PVDF membrane was transferred with proteins and then sealed with the sealing solution of skimmed milk powder. The sealing condition was 80 rpm at room temperature for 2–4 h. Diluted rabbit antihuman LRP (1 : 1,000), rabbit antihuman *β*-catenin (1 : 1,000), rabbit antihuman *β*-actin (1 : 10,000), and rabbit antihuman *α*-tubulin (1 : 10,000) were added and incubated overnight at 4°C. The primary antibody was recovered and washed with Tris-buffered saline/Tween (TBST) three times. The diluted secondary antibody was added and incubated at room temperature for 2 h. The membrane was washed with TBST three times. The ECL protein development kit was used to develop the protein bands of the sample, and the gel imaging system (BIO-RAD, USA) was used for image acquisition and image analysis. The data were standardized with the household-looking genes *β*-actin and *α*-tubulin as an internal reference for LRP5 and *β*-catenin, respectively. All experiments were repeated three times.

### 2.6. Statistical Analysis

SPSS 19.0 was used for statistical analysis of experimental data, and all experimental data were expressed as mean ± standard deviation. Differences between groups were statistically analyzed by one-way analysis of variance, and *P* < 0.05 was considered to be statistically considerable.

## 3. Results

### 3.1. Identification of MG63 Cells

The culture identification of the newly inoculated cells was performed to observe the adherent growth state of the cells during the culture process. In Figure 1, the MG63 cells after three days of normal culture were fully stretched, and the cell morphology was relatively irregular, mostly showing the growth state of a spindle, triangle, or irregular shape, with abundant cytoplasm and obvious nucleolus. After MG63 cells were inoculated on the slides and stained with ALP, the stained cells appeared bluish-purple, and part of the cytoplasm appeared as obvious dark granular. After being stained with Alizarin Red, the cells showed successful stains of the mineralized nodules in MG63 cells.

### 3.2. Titanium Sheet Electron Microscope Scan Pictures

Morphological differences in titanium sheets after different surface treatments were observed by scanning electron microscopy (SEM), as presented in Figure 2. Scratches in the same direction were observed on the surface of group P. The surface of group S presented a nanoscale porous structure, which was irregular in shape and composed of raised trabecular structure.

### 3.3. The Effect of FSS on the Gene Expression of MG63 Osteoblasts on Different Titanium Implant Surfaces

The differences in LRP5 mRNA levels in MG63 cells on different titanium planting surfaces after FSS treatment were detected, and the results were shown in Figure 3. There was no remarkable difference in the level of LRP5 mRNA in MG63 cells between the stressed group and the stationary group (*P* > 0.05). However, the overall expression level of LRP5 mRNA in group *G* was considerably higher than that in group S (*P* < 0.01). The expression level of LRP5 mRNA in each group was the highest at 1 h, and the expression level of LRP5 mRNA in each group was the lowest at 0 h.

The difference in *β*-catenin mRNA levels in MG63 cells on different titanium planting surfaces after FSS treatment was detected, and the results are shown in Figure 4. The expression level of *β*-catenin mRNA in MG63 cells in the stressed group was considerably higher than that in the stationary group (*P* < 0.01). There was no remarkable difference in *β*-catenin mRNA levels in the stationary group at different time points (*P* > 0.05). Except for those at 0 h and 1 h, the expression level of group *G* was always the highest at other time points. Except for those at 2 h and 4 h, the expression level of group S was always the lowest at other time points. The levels of *β*-catenin mRNA in the stressed group were considerably different at different time points (*P* < 0.01). After FSS treatment for four hours, the levels of *β*-catenin mRNA in group P and group S were considerably higher than those in group G (*P* < 0.01).

### 3.4. The Effect of FSS on the Protein Expression of Primary Osteoblasts and MG63 Osteoblasts on Different Titanium Implant Surfaces

The changes in the expression level of LRP5 protein in MG63 cells on different titanium planting surfaces after FSS treatment were detected, and the results are shown in Figure 5. The average LRP5 protein expression level in MG63 cells of the stressed group and the stationary group was considerably different, and the protein expression level of the stressed group was considerably lower than that of the stationary group (*P* < 0.01). Under different FSS treatments, the LRP5 protein expression level of group *G* was considerably higher than that of group P and group S (*P* < 0.05), but there was no remarkable difference between the expressions of group S and group P (*P* > 0.05). The expression levels of each group were high at 0.25 h, 0.5 h, and 1 h. After 4 h of treatment, the expression level of LRP protein in group G was considerably higher than that in group S and group P (*P* < 0.01). The expression level of LRP protein in group S in the stressed group was considerably higher than that in group G and group P (*P* < 0.01).

The changes in *β*-catenin protein expression in MG63 cells on different titanium seeding surfaces after FSS treatment were analyzed, and the results are shown in Figure 6. The difference in the average *β*-catenin protein expression level in MG63 cells of the stressed group and the stationary group suggested that the average *β*-catenin protein expression level in the MG63 cells of the stressed group was considerably higher than that in the stationary group (*P* < 0.01). The expression level of group S was considerably higher than that of group G and group P (*P* < 0.05), but there was no remarkable difference between the expressions of group G and group P (*P* > 0.05). The expression level of *β*-catenin protein in both the stressed group and the stationary group was the lowest at 0 h. Moreover, the expression level of *β*-catenin protein in the three groups of titanium-planted surface MG63 cells under different FSS showed a trend of first increasing and then decreasing over time.

## 4. Discussion

At present, many studies showed that giving corresponding biomechanical stimulation can promote cell proliferation, activation-related cell signaling pathways, and activates the expression of a series of target genes [14–16]. The Wnt pathway plays an important role in the differentiation process of osteoblasts. In this signaling pathway, Wnt protein and its receptors are combined to transmit signals in the cell. The transmission pathways include Wnt/beta-catenin scanning pathway (classical Wnt signaling pathway), Wnt/Ca^2+^ pathway, and Wnt/JNK/Planar cell polarity pathway (PCP pathway) [17, 18]. The main components of the Wnt/beta-catenin scanning signaling pathway are extracellular factor Wnt, transmembrane receptors LRP5/LRP6 and Frizzled, and cytoplasmic protein *β*-catenin [19]. As an important coreceptor of Wnt protein, LRP5 has become a focus for exploring changes in bone density in recent years, and loss of LRP5 function can cause a decrease in bone density [20, 21]. *β*-Catenin is a core member of the Wnt/beta-catenin scanning signaling pathway. When the Wnt signaling pathway is activated, Wnt can interact with Frizzled and LRP5 receptor, and then activate LRP5 and induce axin binding, activate Frizzled and induce Dsh binding. Dsh protein activates the phosphorylation of GSK3*β* and ultimately inhibits the phosphorylation of *β*-catenin [21].

Bone tissue often adapts to changes in mechanical loading through changes in structure and density. In this process, bone cells are the first to perceive changes in bone tissue [22]. Bone cells can transmit these mechanical signals and secrete related signal molecules to regulate the activities of bone-forming cells (osteoblasts) and bone resorption cells (osteoclasts) [23]. It was reported that mechanical stimulation can promote the secretion of Wnt protein [24]. Studies also showed that FSS can activate the expression of *β*-catenin [25]. It has been confirmed that Wnt/beta-catenin scanning signaling pathway is involved in biological processes such as proliferation, differentiation, and metastasis of a variety of cells. Tang et al. [26] confirmed that Wnt/beta-catenin scanning signaling pathway is involved in regulating monoterpene-induced cell proliferation inhibition. Ma et al. [27] showed that *β*-catenin can activate the expression of downstream target genes that regulate the cell cycle, and thus participate in the proliferation pathway of chondrocytes. Exploration of the effect of FSS stimulation on the expression levels of LRP5 and *β*-catenin mRNA and protein in cells showed that the FSS of 12 dynes/cm^2^ can promote the expression level of *β*-catenin mRNA and protein without affecting the expression level of LRP5 mRNA but can inhibit the expression level of LRP5 protein. Studies pointed out that the expression of LRP5 mRNA and protein in MG63 cells on the titanium surface was inhibited after sandblasting and acid-base treatment and the expression of *β*-catenin was promoted. The surface properties of titanium after sandblasting and acid-base treatment can promote the proliferation and differentiation of MG63 cells, and this effect can be achieved by activating the Wnt/beta-catenin scanning signaling pathway. Wang et al. researched and analyzed the surface and smoothness of nanostructured titanium, and it was revealed that the apoptosis rate of upper MG63 cells was low, and there was no remarkable difference between the groups. However, the *β*-catenin pathway was obviously activated in the cells on the surface of nanostructured titanium and the osteogenic activity was enhanced [28]. In summary, the titanium surface can promote the proliferation of osteoblasts by regulating the transcription levels of LRP5 and *β*-catenin in the Wnt/beta-catenin scanning signaling pathway after FSS and sandblasting acid-base treatment.

## 5. Conclusion

In summary, 12 dynes/cm^2^ FSS and sandblasting acid-base treatment on the titanium surface can promote the expression of *β*-catenin and inhibit the expression of LRP5, which in turn plays a role in promoting osteoblast proliferation. However, this work only explores the effect of FSS on cell proliferation in vitro and the expression levels of LRP5 and *β*-catenin in the Wnt/beta-catenin scanning signaling pathway. The proliferation activity and apoptosis rate of osteoblasts after different surface treatments were not detected in this study. In the follow-up, it is necessary to further establish corresponding animal models to verify the regulatory mechanism in vivo, and the Wnt/beta - catenin scanning pathway inhibitors shall be added to explore the effect of this pathway on the proliferation and differentiation level, osteogenesis ability of osteoblasts. In conclusion, this study initially explores the mechanism of cellular mechanics signal transduction related to the implant-bone interface, which lays the foundation for further research on the cell biomechanics of the implant cell interface.

## Figures and Tables

**Figure 1:** Morphology and staining observation of MG63 cells.

**Figure 2:** SEM observation of titanium sheet surface with different surface treatments (×20,000).

**Figure 3:** LRP5 mRNA detection results of MG63 cells. (a) 0 dynes/cm^2^ stationary group; (b) 12 dynes/cm^2^ FSS group; compared to group G, ^*∗*^*P* < 0.05 and ^*∗∗*^*P* < 0.01.

**Figure 4:** Detection results of *β*-catenin mRNA in MG63 cells. (a) 0 dynes/cm^2^ stationary group; (b) 12 dynes/cm^2^ FSS group; compared to group G, ^*∗*^*P* < 0.05 and ^*∗∗*^*P* < 0.01.

**Figure 5:** Results of detection of LRP5 protein expression in MG63 cells. (a) Western blot bands; (b) 0 dynes/cm^2^ stationary group; (c) 12 dynes/cm^2^ FSS group; compared to group G, ^*∗*^*P* < 0.05 and ^*∗∗*^*P* < 0.01.

**Figure 6:** Detection results of *β*-catenin protein expression in MG63 cells. (a) Western blot bands; (b) 0 dynes/cm^2^ stationary group; (c) 12 dynes/cm^2^ FSS group; compared to group G, ^*∗*^*P* < 0.05 and ^*∗∗*^*P* < 0.01.

**Table 1:** Quantitative primer sequences.

Gene	Primer (3′⟶5′)
LRP5-F	TTCATCCACCGTGCCAAC
LRP5-R	TGTCCAGTACAGAGTGTCCC
*β*-Catenin-F	AAGGTGCTATCTGTCTGCTC
*β*-Catenin-R	TGACTTGGATCTGTCAGGTG

## Data Availability

The data used to support the findings of this study are available from the corresponding author upon request.
